# An Intelligent Analysis Model in the Environment of Regional Economic Development and Regional Economic Differences in China Using Big Data Analysis Technology

This article has been retracted.

**DOI:** 10.1155/2022/8935743

**Published:** 2022-08-31

**Authors:** Junyin Luo

**Affiliations:** School of Economics, Beijing Technology and Business University, Beijing 100048, China

## Abstract

The current and long-term regional economic imbalance in China requires ongoing attention. To ensure the balanced development of China's renewable energy, it is therefore important to examine the causes of the differences in China's renewable energy from a variety of perspectives. The spatial distribution pattern and characteristics of China's per capita GDP (gross domestic product) from 2012 to 2021 were examined in this study using the exploratory spatial data analysis tool. In addition, it conducts an empirical investigation into the spatial spillover effect of RED and the manufacturing agglomeration in China (regional economic development). The findings indicate that in the eastern region, the total backward link value of the feedback effect of 17 industrial sectors is 0.8524, and in the central region, the value is 0.8139. The real per capita GDP of neighboring provinces will increase by 0.118% for every 1% increase in manufacturing agglomeration level. According to the overall ranking, China's RED level is very uneven due to a number of factors. We should direct and encourage the manufacturing industry to congregate in various regions, optimize the spatial pattern of manufacturing industry agglomeration, and fully exploit SSE in order to promote China's RED and reduce the difference in RE.

## 1. Introduction

As an economic phenomenon, the RED (regional economic development) difference is the end result of a variety of factors, including geographic location, resource endowment, infrastructure, cultural and historical environment, policy system, and others. The effects of various factors, however, frequently vary between regions and time periods [1]. China's regional economies (RE) gap is widening, RE is insufficient and poorly coordinated, and the regional industrial structure is unjust. These factors lead to inequality, which impedes China's economic development and makes it more likely that issues will arise that threaten social and political stability. The so-called cross-regional SE (spillover effect), which first appeared in China's RED, has been a major contributor to other regions' rapid economic development. China's obvious development gaps between different scales and regions, which have emerged as the primary manifestation of the main social contradiction “imbalance” in the new era, are despite the country's gradual strengthening of its comprehensive national strength and the acceleration of its modernization process. The correct definition of China's high-quality economic development now centers on closing the regional development gap, and in the modern era, this is a crucial step in resolving serious social conflicts [2].

The disparity in regional development is significant on a global scale, and the use of renewable energy varies widely. There are variations in the rates of economic growth among regions, regardless of whether the countries are developed or developing, capitalist or socialist. According to Gómez‒Zaldívar et al., China has clearly made progress in comparison to other underdeveloped nations as the gap in relative income between its provinces and regions has shrunk [3]. The gap between the three major areas is much smaller than that indicated by per capita GDP, according to Chen's per capita net income for farmers and per capita disposable income in urban areas (gross domestic product). He believes that China's regional differences are within an acceptable range because the difference is largely due to differences in urbanization levels [4]. Zhou et al. used the reciprocal of the Herfindal index as the measurement index of the scope economy to calculate the Herfindal index of 19 cities. The findings demonstrate that whether an economy has the potential for divergence depends on the size of cities and the transportation costs of industrial development [5]. Knowledge transfer and localized information, according to Hong et al., not only helped cities form economic agglomerations but also fueled their expansion economically [6]. This causes confusion in the RED model research. Due to the RED model's rapid evolution and transformation against the backdrop of economic globalization, the RED model now exhibits new traits and trends.

The coordinated development of renewable energy is being given more attention by the central and local governments as China's economy transitions to a new normal, while also placing an emphasis on the quality of economic development, particularly how to use the leverage effect of regional economic development to promote economic development in underdeveloped areas [7]. Gain an understanding of the general development trend, investigate the issues that prevent China from developing renewable energy in a coordinated manner, and conduct in-depth investigation and analysis to various degrees. China is moving toward a coordinated development of renewable energy. From a practical standpoint, through the empirical analysis of the benefits and channels of various types of REDSE in China, the characteristics, modes, and directions of regional economic relations in China are thoroughly investigated, which can provide theoretical guidance for the direction. Research the inter-regional economic cooperation and China's policy direction for renewable energy, and offer theoretical guidance for the inter-regional economic cooperation and China's policy direction for renewable energy.

Innovation of research as:

1. This paper makes an empirical test on the growth SE of national economic development zones by using a variety of different model methods and analyzes the difference in growth SE of different economic benefits of national economic development zones, as well as the difference of growth SE of national economic development zones in different locations, different levels of technological innovation and different regions.
2. For many renewable energy units with complete functions, relevant scholars often ignore the correlation between the region and the surrounding economy in their research, and the conclusions drawn from this are often unreasonable in explaining the phenomenon of the real economy. In order to avoid the abovementioned problems, this paper brings spatial factors into the economic growth model and improves the explanatory power of the model conclusions.

## 2. Related Work

### 2.1. Research Status of RE Differences

Currently, China is deepening its supply-side structural reforms and continuously enhancing the leadership position of innovation in science and technology. China's economy is also struggling with uneven and insufficient growth at the same time. The ongoing expansion of macroaggregates and the widening gap between microregions are characteristics of China's economic development. The introduction of relatively more high-tech jobs in the eastern region following the reform and opening up is the primary cause of the economic gap between it and the central and western regions. The regional development gap is further widened as labor mobility restrictions are relaxed and skilled labor moves from the central and western regions to the eastern regions.

Tong et al. pointed out that China's unbalanced development strategy and measures to restrict population mobility are the keys to the income gap between teaching and research groups [8]. Zhou et al. decomposed the Sill coefficient of GDP and total industrial output value and concluded that although the differences between coastal areas narrowed, the differences between coastal areas and inland areas were constantly expanding [9]. Brekke pointed out that the perfect property right system is the key driving force of China's economic development, especially since the private economy will gradually become the main body of China's economic development [10]. Ding et al. put forward the dynamic mechanism model of regional development model innovation through induction and believed that natural factors, historical factors, government factors, and residents factors were the foundation and driving force of regional development model innovation. At the same time, these factors will lead to the convergence and difference of different development models [11].

Astafyeva analyzed RE by using the per capita gross industrial and agricultural output value as an index. The selected index is relatively simple in calculation and convenient to use, but its representativeness is not strong and it is relatively single [12]. Dotti and Spithoven, through the analysis of China's regions, think that the influence of geographical factors on the growth of China's coastal economy is more lasting than that of policies. At the same time, it is also found that the household registration system, trade protection, and bank lending policies will further widen the gap of RED [13]. Tang et al., based on spatial econometrics, analyzed the standards of economic convergence and extended them. All cities at the prefecture level and above in China are qualified to discuss economic convergence [14].

### 2.2. SSE and Economic Growth Research

SSE (Space Spill Effect) is the space economy of SE. In early classical economics, spatial economics was used to describe the formation and development of industrial locations. Space economy is considered as a complex spatial form of economic activity. Industrial agglomeration often leads to SSE, and the existence of this effect is mainly due to the integration and optimization of spatial material elements and the increase of labor and capital operation density. This external effect, which crosses the boundaries of one or more economies and radiates and promotes the development of many economies at the same time, constitutes the basic connotation of the SSE.

Ustaoglu et al. defined knowledge spillover as the phenomenon that the knowledge owned by foreign enterprises was acquired by local enterprises without formal transfer of foreign enterprises [15]. There is an essential difference between knowledge spillover and knowledge diffusion. Spillover is an individual form of knowledge diffusion, that is, information is obtained through communication and interaction between subjects, and the receiver who enjoys the intellectual achievements does not give the knowledge innovator enough economic compensation or pay the corresponding full cost. Bennett et al. put forward that culture, history, system, and other elements are generally taken seriously in new economic geography, and the corresponding consideration indicators will be added to measure them in the research [16]. Sebastian further analyzed the role of basic public services in RED. Through analysis, they believed that the agglomeration degree of regional pattern depends on the equalization level of public services in the region. The higher the equalization level, the more dispersed the overall layout of RE will be [17].

Wang and Wang pointed out that, unlike ordinary commodities, because knowledge is widely disseminated and can produce obvious positive SE, the knowledge produced by any manufacturer can improve the productivity of the whole society [18]. Fu puts forward technology SE and thinks that demonstration, imitation, and dissemination are the increasing functions of technological information differences. Competition is influenced by the market characteristics of multinational companies and local manufacturers, and technology SE can be produced through demonstration, imitation and dissemination, and competition [19]. Fang and Fang tried to further divide the technology gap, suggesting that too big or too small a technology gap is not conducive to local enterprises' access to technology SE [20].

## 3. Methodology

### 3.1. RE Spatial Structure Evolution and Inter-Regional Economic Relations

The analysis of the regional development gap from the standpoint of input and factor allocation, focusing on labor force size, human capital disparity, capital scarcity, technological capability, and factor allocation efficiency, is the main objective of the determinism of economic growth factors. Due to the rapid growth China's economy, the financial and logistics sectors have emerged as crucial engines for the country's continued economic expansion. The growth pole's construction will have a detrimental effect on the surrounding areas as well. The high-quality talent and abundant resources in the surrounding areas will be drawn to the center of the growth pole, which will weaken their ability to innovate and competitive advantage to some extent, slowing down the rate of economic growth.

The lack of capital, advanced technology, and managerial skills are just a few of the constraints that developing nations must contend with because of their outdated economies and technologies. China's terrain has a stepped distribution, high in the west and low in the east. In the aforementioned ways, the central and western regions, particularly the western ones, are clearly inferior to the eastern ones. Furthermore, it is challenging to achieve meaningful results for large-scale economic development and construction due to traffic limitations. Incredibly quickly. In this situation, economically and technologically underdeveloped regions should work on enhancing their capacity for acceptance and learning while focusing on raising the rate at which seed delivery technology is adopted by the general public.

For any region, the topic of economic development always occupies the central position, which is the basis for solving the problems of social and economic development. Therefore, RED is also the core research content of RE and economic geography. Economic development originates from the professional division of labor, which promotes the improvement of labor productivity, and then promotes the economic development of a country. The elements of economic development also include organizational management, technological innovation, economies of scale, and structural changes. Subsequently, people further expanded the elements of economic development into material capital, human capital, natural resources, infrastructure, technology, and system. In the process of spatial structure evolution of renewable energy, there are many kinds of interactions among regions, among which the inter-regional flow of production factors and the inter-regional trade of products are the two most important inter-regional economic ties.  Figure 1 summarizes the main modes of regional interaction.

Labor force migration between regions and capital flow between regions make up the inter-regional flow of production factors. The transfer and spread of inter-regional industries are reflected in the inter-regional flow of production factors. Production increases in scope. The state of inter-regional industrial links is reflected in the flow of goods between regions. The interaction of various regional factors is important for economic growth and development, but so are the external effects of those factors and product flows.

In the course of economic development, industrial agglomeration is a typical phenomenon that manifests itself in various nations, cities, or regions. It consistently supports and ensures the development of China's national economy as a key component of industrial economic development. In order to measure and analyze the overall agglomeration level of China's manufacturing industry, this paper primarily uses the GC (Gini coefficient) position. It uses the following calculation formula:

(1) $$\begin{array}{c} G_{i}=\frac{1}{2n^{2}\delta }\sum_{a}\sum_{b}\left|\frac{x_{ia}}{X_{i}}-\frac{x_{ib}}{X_{i}}\right|, \end{array}$$

where *G*_*i*_—GC location; *n*—The number of regions, *n* in this paper is the 31 provinces in my country; *δ*—*i* the average number of employees of the industry in each province; *x*_*ia*_, *x*_*ib*_—Industry *i* employment in Provinces *a* and *b*, respectively; *X*_*i*_—The total number of employed people in *i* industry.

The value range of *G*_*i*_ is [0,1], and the greater the location *G*_*i*_, the higher the degree of industrial agglomeration.

GC can decompose the total income gap between different subincome gaps. However, this method has its own limitations, and it cannot be used to decompose the total economic gap among different groups (or regions). The relationship between the total income *G* and its various sub-income can be written as:

(2) $$\begin{array}{c} G=\sum \left(U_{i}\times C_{i}\right), \end{array}$$

where *U*_*i*_, *C*_*i*_ is the share and concentration ratio of item *i* income in total income.

The total output ultimately depends on the complicated intermediate production process determined by the technical and economic structure of the production system. The inter-regional input-output table established by the input-output analysis technology mainly reveals the inter-regional industrial relevance, thus analyzing the production-induced effect and industrial indirect effect brought by the inter-regional demand relationship. From the practical application, the basic form of the demand attraction model in the input-output analysis is as follows:

(3) $$\begin{array}{c} \Delta X={\left(I-A\right)}^{-1}\Delta Y. \end{array}$$

Among them, Δ*Y*—Represents the final demand change determined by factors outside the system; (*I* − *A*)^−1^—Leontief health matrix, which is a parameter in the system; Δ*X*—The change of total output determined by exogenous variables and system parameters.

This paper adopts the financial development indicators of most domestic scholars and measures financial development mainly from two angles: scale and efficiency. The scale of financial development is expressed by the ratio of total deposits and loans of regional financial institutions to GDP, namely:

(4) $$\begin{array}{c} F_{\text{index}}=\frac{FI_{\text{total deposits}}+FI_{\text{Total loan amount}}}{GDP}. \end{array}$$

Among them, *F*_index_—Financial indicators; *FI*_total deposits_—Total deposits of financial institutions; *FI*_Total loan amount_—Total loans of financial institutions The efficiency of financial development is the ratio of total deposits and loans of regional financial institutions.

Opening to the outside world and attracting foreign investment is another important factor in China's rapid economic growth. The inflow of foreign capital into China not only brings more capital but also more advanced technical means and management experience, which accelerates the pace of China's integration into globalization, thus accelerating the pace of China's economic construction. In addition, the gathering of foreign capital promotes capital accumulation, provides strong financial strength for regional development, injects new impetus into scientific and technological research and development, leads the host country to produce more advanced products, and makes use of domestic and foreign high income to flow into the terminal market. The abovementioned influencing mechanism and driving path are shown in Figure 2:

### 3.2. Mechanism Analysis of SSE

The idea of SSE is comparable to the concept of externality in western economics, which states that an organization's actions not only affect them directly but also may have an equal or opposing effect on nearby organizations. SSE denotes the idea that an economy's economic activity will not only have an effect on its own economy but will also have an equivalent effect on its neighboring economies. Large companies' financing issues have been resolved thanks to the growth of the stock market, which has also reduced moral hazard and transaction costs for company managers, enhanced corporate governance capabilities, and boosted economic growth. The new institutional economics school holds that since knowledge is easily imitated, even though businesses acquire knowledge quickly, it can still be quickly imitated by rival businesses. As a result, businesses must take measures to protect themselves.

In the investigation of this paper, we will focus on the SE of China's provincial economic growth, and analyze the spatial related characteristics and economic growth factors of 31 provinces in China by spatial statistical methods and spatial econometric techniques. The existence of spatial correlation will definitely be reflected in SSE measurement. Combined with the theory of economic growth, this paper describes the dynamic relationship between the national economic development zone and the parent cities outside the zone in detail by adopting a relatively static analysis method. Considering the complexity of real economic behavior, after analyzing the basic model, we can draw richer conclusions by relaxing the analysis assumptions.

In the long run, the inflow of transportation infrastructure investment expands the scale stock of transportation infrastructure and then drives the growth of total factor productivity of the manufacturing industry through the direct promotion effect of scale stock and SSE. As shown in Figure 3.

The expansion and promotion of cross-regional trade of people and goods facilitate the transfer of knowledge and technology. Transportation infrastructure development and improvement are therefore beneficial. The growth and development of transportation infrastructure results in increased regional accessibility and ongoing reductions in transportation costs. As a result, the protection tax rate is decreased, technology expansion industries are eliminated, and the technical effectiveness of the surrounding RE is improved. The creation and upkeep of transportation infrastructure will act as a lubricant, lessen resistance to the flow of resource components, and encourage the initial state of allocation to get closer to the equilibrium point of optimal allocation. The aforementioned influencing mechanisms have a clear logical and progressive relationship with one another. In particular, increasing export comparative advantage can hasten regional market integration and support the clustering of economic activities, and regional market integration can support these effects even more. In order to accurately and completely assess the contribution of transportation infrastructure to economic growth or productivity growth, the SSE for transportation infrastructure is included in the measurement framework of the growth effect of transportation infrastructure.

In the short term, because capital cannot flow freely, the labor force can be transferred to places with higher marginal returns by changing their work forms. Therefore, in the short term, the flow of the labor force will change the marginal output level of production factors in national economic development zones and mother cities outside the zones. Therefore, it is necessary to use the local indicators of spatial correlation to analyze the local characteristics of spatial correlation. The local Moran's I index is the main index to measure the regional spatial local autocorrelation:

(5) $$\begin{array}{c} I_{i}=Z_{i}\sum_{j=1}^{n}W_{ij}Z_{j}, \end{array}$$

where *Z*_*i*_, *Z*_*j*_ represents the observed value of *i*, *j* region, in this paper, it is GDP per capita, *n* is the number of regions, and *W* is the spatial weight matrix. This index measures the degree of correlation between the *I*-th region and other surrounding regions.

The unbalanced index *E* is used to measure the unbalanced overall pattern of regional GDP distribution [20], and the calculation formula is as follows:

(6) $$\begin{array}{c} E=\sqrt{\frac{{\sum_{i=1}^{n}\left[\left(\sqrt{2}/2\right)\left(X_{i}-Y_{i}\right)\right]}^{2}}{n}}, \end{array}$$

where *n* is the total number of research units; It indicates the GDP and area ratio of *X*_*i*_, *Y*_*i*_ city *i* to the total.

EMD (emotional mode decomposition) decomposes the time signal *X*(*t*) into a series of IMF‚ (Intrinsic Mode Function‚). For the time series *f*(*t*), if there is only one fluctuation with scale *σ* in the neighborhood (*t*_0_ − *σ*, *t*_0_+*σ*) of a certain point *t*_0_, the local average of *f*(*t*) can be expressed as:

(7) $$\begin{array}{c} I_{\sigma }=\int_{t_{0}-\sigma }^{t_{0}+\sigma }f\left(t\right)\text{dt}. \end{array}$$

The area enclosed by the time axis in one cycle of fluctuation is zero, which is the symmetry requirement of *I*_*σ*_⟶0 relative to the time axis.

In this paper, the absolute *β* convergence equation of RE is taken as the starting point of analyzing the problem. Firstly, the general absolute *β* convergence model is set as follows:

(8) $$\begin{array}{c} \ln=\alpha \frac{\left(Y_{it+k}/Y_{it}\right)}{k}+\beta \;\ln\left(Y_{it}\right)+\mu_{i},\;i=1,2,n, \end{array}$$

where *Y*_*it*+*k*_ represents the actual per capita income level in *t*+*k* year, and *Y*_*it*_ represents the actual per capita income level in *t* year of the *i* th region, so ((*Y*_*it*+*k*_/*Y*_*it*_)/*k*), as the dependent variable of the model, represents the average growth rate of the *i* th region in *k* years.

Conditional *β* convergence model is to add control variables on the basis of the abovementioned formula, which can be specifically expressed as follows:

(9) $$\begin{array}{c} \ln\frac{\left(Y_{it+k}/Y_{it}\right)}{k}=\alpha +\beta_{1}\ln\left(Y_{it}\right)+\beta_{2}X_{ij+k}+\mu_{i},\;i=1,2,n, \end{array}$$

*X*_*ij*+*k*_ represents those variables that can control the stable state.

If all regions are divided into *G* groups in a certain way, the Thiel coefficient can be decomposed as follows:

(10) $$\begin{array}{c} I\left(o\right)=\sum_{g=1}^{G}p_{g}I{\left(o\right)}_{g}+\sum_{g=1}^{G}p_{g}\text{log}\frac{p_{g}}{v_{g}}, \end{array}$$

where *v*_*g*_ represents the share of income of Group *g* in the total income, and *p*_*g*_ represents the share of population of Group *g* in the total population. Therefore, the overall regional income difference can be decomposed into the sum of the differences within and among the three major zones.

## 4. Experiment and Results

### 4.1. Exploratory Spatial Analysis of Economic Growth

The relationships between the various regions in China's vast country frequently have unique characteristics. In comparison to other regions, East China's development of an economic, political, cultural, social, and ecological civilization is more dynamic. These areas serve as the government's primary area of focus and influence, which is a reflection of its strong governance capacity. The eastern region and other regions have very different levels of governance. Since human activities have finite amounts of energy, resources, and capacity, learning will always require a financial investment in the form of time and resources. However, because of the intricate division of labor, it is impossible for local subjects to become fully knowledgeable in all fields of expertise. Knowledge can therefore only be held by various people in a decentralized manner; it cannot be held in a centralized manner.

The agglomeration effect gradually emerges and takes over when the factors come together to a certain extent, leading to uneconomical agglomeration, a slowing down of economic growth, a beginning of the flow of the labor force back, an acceleration of economic growth in underdeveloped areas, and a narrowing of regional disparities. Additionally, some mechanisms are in place to reduce the growing regional disparities. We first examine the characteristics of economic growth's spatial dependence before applying spatial model analysis.  Table 1 lists the global Moran's I index and its meaning.

It can be seen that the values of Moran's I index are all between 0.23 and 0.27. According to the value of P, Moran's I index is significant at the test level of 1%, which indicates that economic growth has a certain positive spatial correlation, and the spatial correlation of economic growth has been kept at a stable level.

The distribution of production factors across countries and regions is unbalanced as a result of natural conditions, natural resources, traffic conditions, the economic and social environment, and other factors. This results in differences in the relative prices of production factors. Prices of essential goods, which then encourage inter-regional trade. Analysis of a region's good development and formation of a unique RED model is aided by knowledge of its regional competitive advantage. Demand quality from domestic consumers is more significant than demand volume. Firms are compelled to continuously innovate, improve, and boost their competitiveness by the tough market demand and picky consumers.

By combining 78 groups of two provinces each year according to the relative price changes of each province, the annual relative price changes of each province can be obtained. The results show that in the sample period, the market segmentation degree of each province tends to expand first and then shrink, but the market segmentation degree and the variation range of each province are quite different. The results are shown in Figure 4.

It can be found that the market segmentation degree of Ningxia, Heilongjiang, Fujian, Hebei, Liaoning, and Shaanxi shows a downward trend in general, indicating that the market segmentation degree of these provinces has steadily declined with the passage of time; the market segmentation degree of Shanxi, Yunnan, Gansu, and Qinghai is on the rise as a whole, which shows that the market segmentation degree of these provinces has been steadily rising.

### 4.2. REDSE Analysis of Inter-Regional Product Flow

Cross-regional SE refers to the impact of renewable energy development on another RED. From the perspective of cross-regional entry and exit, it reflects the change of the final industry in one region, which leads to the production of the total output in another region. This work measured the intra-regional multiplier effect, inter-regional SE effect, and feedback effect in the eastern and central regions of China, and the results are shown in Figures 5–7.

In the eastern region, the total backward linkage value of the feedback effect of 17 industry sectors is 0.8524, while the corresponding value in the central region is 0.8139, as can be seen in Figure 7. Economically speaking, it means that while the final demand in the eastern region increases simultaneously by 1 unit in each industrial sector, the corresponding value in the central region is 0.8139 units. Because the SE values between the eastern and central regions are so low, the feedback effect values of the two regions are both quite small. The two regions' combined feedback effect in various industries exhibits similar industrial traits to SE.

Manufacturing of nonmetallic minerals, wood products, furniture, and the provision of electricity, hot water, gas, and water are the largest SEs from the eastern to the central regions. The fact that the third industry is also fairly large and resource-intensive demonstrates how heavily the eastern part depends on the resources of the central part. The products of labor-intensive industries with clear advantages in the eastern region, in addition to the technology-intensive industries in the eastern region, are heavily reliant on the western region. Similar to one another, the two regions' high-SE industries are primarily concentrated in the production of transportation equipment, machinery, castings and metal products, and electronic and electrical equipment. The industrial characteristics are similar and the regional feedback effect between the two regions is very small.

### 4.3. SSE Analysis of Manufacturing Agglomeration and RED

According to the results of the spatial autocorrelation test, it can be found that there is a very significant spatial autocorrelation in China's RED, and a suitable spatial econometric model can be established to analyze SSE and RED in manufacturing clusters. Generally speaking, when the sample regression analysis is limited to some specific individuals, it is more appropriate to adopt the fixed effect model, so this paper adopts the fixed effect model for analysis [13]. The decomposition results are shown in Table 2. Among them, the direct effect represents the influence of each explanatory variable on the economic growth of this province, and the indirect effect represents the influence of each explanatory variable on the economic growth of neighboring provinces. The total effect is the sum of direct effect and indirect effect, which represents the total influence of each explanatory variable on economic growth.

The direct impact coefficient of manufacturing agglomeration in RED is 0.047, but it has not passed the significance test. This shows that manufacturing agglomeration has a positive effect on the economic growth of the whole province. For every 1% increase in manufacturing agglomeration level, the real per capita GDP of neighboring provinces will increase by 0.118%. With a strong SSE, RED can be effectively promoted in neighboring provinces.

The labor input has a negative direct impact of −0.203, a negative indirect impact of −0.562, and a negative total impact of −0.782, all of which pass the 1% significance test. It demonstrates that labor input not only has a detrimental effect on this province's economic growth but also restrains the economic growth of nearby provinces. The primary engine of RED no longer involves labor input. Government policy support has a markedly negative spatial effect on RED, indicating that it restricts the development of renewable energy and, to some extent, prevents effective resource allocation from occurring in the public finance budget. Local governments may also implement local protectionist policies to safeguard the growth of renewable energy in the area, which will have a certain detrimental effect on RED, driven by local interests.

In this section, 12 samples of national economic development zones in 2012–2021 are selected as input indicators, including capital input and labor input of foreign parent cities, and GDP as output indicators. When calculating the efficiency index of each source city outside the area, the average value of each year is used as the evaluation index, and the results are shown in Figure 8 below.

It can be seen that the total factor productivity of Qinhuangdao, Daya Bay in Huizhou, and Tianjin is relatively high. The technical efficiency, technological progress, pure technical efficiency, scale efficiency, and total factor productivity of Qinhuangdao are all greater than 1. The technical efficiency, pure technical efficiency, and scale efficiency of Daya Bay in Huizhou are all 1, which shows that the production scale of the three cities is relatively reasonable, the technical equipment is more advanced, and the input ratio and factor combination are relatively optimized. At present, there is large population mobility in various regions of China, and the per capita economic development is generally unbalanced. This imbalance has hindered China's economic growth and social progress.  Figure 9 shows the average score of RE level in China.

It can be seen the top three are Beijing, Shanghai, and Tianjin. The comprehensive scores of the three regions are relatively high, indicating that their economic development level is very high, while other RED levels are generally even lower. Guizhou, which ranks first from the bottom, has a difference of 2.8 points, more than 4 times. It can be seen that the gap between them is particularly obvious. Judging from the overall ranking, China's RED level is very uneven due to various factors.

According to the state of the economy right now, there are still systemic issues preventing the central and western regions as well as the entire nation's economic development. We should hasten state-owned enterprise reform, maximize the nonpublic economy's contribution to the nonpublic economy, fully exploit the vitality of various ownership economies, and support the overall growth of state-owned enterprises in order to achieve the best ownership structure. We should also expand our horizons and raise the caliber of our own work at the same time. At the same time, we should improve service areas, increase investment attraction, and improve our opening to the outside world. Create a service sector that adapts to the times, pursues emerging trends, and places a premium on the growth of the service outsourcing sector.

## 5. Conclusions

In the stage of high-quality development, closing the regional development gap is both a key component of China's high-quality economic development and one of the major challenges facing future social development. This study compares China's RED and RE based on SSE, looking at 31 Chinese provinces from the perspective of spatial geography from 2012 to 2021. Following are the key conclusions: the central region's equivalent value in terms of backward linkage is 0.8139, and the eastern region is 0.8524 for the feedback effect of 17 industrial sectors as a whole. The economic significance is that the final demand would rise by one unit simultaneously in the eastern region of each industrial sector did so, compared to 0.8139 units in the central region. Manufacturing agglomeration's 0.047 direct impact coefficient in RED did not pass the significance test. This demonstrates that the economic development of the entire province benefits from manufacturing agglomeration. China's RED level appears to be very uneven overall based on a number of factors, according to the ranking.

## Figures and Tables

**Figure 1:** Regional economic ties.

**Figure 2:** The mechanism of financial agglomeration affecting RED.

**Figure 3:** Theoretical analysis framework.

**Figure 4:** Ranking status of market segmentation degree in each province and market.

**Figure 5:** Intra-regional multiplier effect.

**Figure 6:** Inter-regional SE.

**Figure 7:** Inter-regional feedback effect.

**Figure 8:** Total factor productivity of mother cities outside each district.

**Figure 9:** RE: level per capita score in China.

**Table 1:** Test results of Moran's I index of economic level.

Year	Moran's I	*P* value
2012	0.236	0.006
2013	0.266	0.009
2014	0.241	0.007
2015	0.268	0.006
2016	0.261	0.008
2017	0.255	0.007
2018	0.251	0.008
2019	0.267	0.008
2020	0.249	0.011
2021	0.268	0.009

**Table 2:** Model spatial effect decomposition.

Variable	Direct effect	Indirect effect	Total effect
Core explanatory variable	0.047 (1.683)	0.118^*∗*^ (1.638)	0.168^*∗∗*^ (1.983)
Labor input	−0.203^*∗∗∗*^ (−4.335)	−0.562^*∗∗∗*^ (−3.214)	−0.782^*∗∗∗*^ (−4.335)
Fixed-asset investment	0.052^*∗∗*^ (2.238)	0.036 (0.605)	0.086 (1.427)
Technical innovation	0.096^*∗∗∗*^ (5.601)	−2.986^*∗∗∗*^ (−7.248)	−0.186 (−4.258)
Infrastructure construction	0.081^*∗∗∗*^ (2.936)	0.008 (0.103)	0.086^*∗∗∗*^ (1.036)
Urbanization	0.328^*∗∗∗*^ (4.016)	−0.639^*∗∗∗*^ (−3.415)	−0.225 (−1.428)
Degree of opening to the outside world	0.047^*∗∗∗*^ (0.046)	0.017 (0.568)	0.055^*∗∗*^ (1.768)
Government policy support	−0.136^*∗∗∗*^ (−2.862)	−2.418^*∗∗∗*^ (−3.263)	−0.369^*∗∗∗*^ (−4.258)

*Note.* ^*∗*^, ^*∗∗*^ and ^*∗∗∗*^ represent the significance level of 0.1, 0.05, and 0.01, respectively. The numbers in brackets are the *t* values of the corresponding variable coefficients.

## Data Availability

The data used to support the findings of this study are included within the article.

## References

[1] Liu X. (2018). Dynamic evolution, spatial spillover effect of technological innovation and haze pollution in China. *Energy & Environment*.

[2] Torres-Preciado V. H., Polanco-Gaytan M., Tinoco-Zermeno M. A. (2017). Crime and regional economic growth in Mexico: a spatial perspective. *Papers in Regional Science*.

[3] Gómez-Zaldívar M., Fonseca F. J., Mosqueda M. T., Gómez-Zaldívar F. (2020). Spillover effects of economic complexity on the per capita gdp growth rates of mexican states, 1993-2013. *Estudios de Economia*.

[4] Zeng C. (2019). Spatial spillover effect on land conveyance fee—a multi-scheme investigation in wuhan agglomeration. *Land Use Policy*.

[5] Zhou B., Wen Z., Sutherland I., Lee S. K. (2022). The spatial heterogeneity and dynamics of tourism-flow spillover effect: the role of high-speed train in China. *Tourism Economics*.

[6] Hong J., Gu J., He R., Wang X., Shen Q. (2020). Unfolding the spatial spillover effects of urbanization on interregional energy connectivity: evidence from province-level data. *Energy*.

[7] Bi Y. (2017). Research and simulation of prediction model of regional economic development potential based on svm method. *Boletin Tecnico/Technical Bulletin*.

[8] Tong X., Li X., Tong L., Chen K. (2019). Research of spatial and temporal evolution mechanism and countermeasures of haze spatial pattern in China: visual field based on dynamic evolution and spatial agglomeration. *Advances in Meteorology*.

[9] Zhou Y., Kong Y., Sha J., Wang H. (2019). The role of industrial structure upgrades in eco-efficiency evolution: spatial correlation and spillover effects. *Science of the Total Environment*.

[10] Brekke T. (2021). What do we know about the university contribution to regional economic development? a conceptual framework. *International Regional Science Review*.

[11] Ding X., Billari F. C., Gietel-Basten S. (2017). Health of midlife and older adults in China: the role of regional economic development, inequality, and institutional setting. *International Journal of Public Health*.

[12] Astafyeva O. V., Astafyev E. V. (2018). Features of the regional economic systems development with a mono-branch focus. *Management Science*.

[13] Dotti N. F., Spithoven A. (2018). Economic drivers and specialization patterns in the spatial distribution of framework programme’s participation. *Papers in Regional Science*.

[14] Tang Z., Zhang Z., Zuo L., Wang X., Hu S., Zhu Z. (2020). Spatial econometric analysis of the relationship between urban land and regional economic development in the beijing–tianjin–hebei coordinated development region. *Sustainability*.

[15] Ustaoglu E., Lavalle C., Boris P. (2017). Examining lag effects between industrial land development and regional economic changes: The Netherlands experience. *PLoS One*.

[16] Bennett M. M., Smith L. C. (2017). Using multitemporal night-time lights data to compare regional development in Russia and China, 1992–2012. *International Journal of Remote Sensing*.

[17] Sebastian J., Jlich, Regional, Economics & Development (2017). Towards a local-level resilience composite index: introducing different degrees of indicator quantification. *International Journal of Disaster Risk Science*.

[18] Wang C., Wang X. (2017). Research on prediction model and coordinated development of regional economic development potential. *Boletin Tecnico/Technical Bulletin*.

[19] Fu D. (2017). Research on the differences of regional economic development model and related factors based on data mining statistical analysis. *Boletin Tecnico/Technical Bulletin*.

[20] Fang Y., Fang S. (2017). A simulation study on the prediction model and general path of regional economic development potential based on panel model. *Revista de la Facultad de Ingenieria*.

